This article has been retracted.

# New Opportunities, Challenges, and Applications of Edge-AI for Connected Healthcare in Internet of Medical Things for Smart Cities

**DOI:** 10.1155/2022/2950699

**Published:** 2022-02-23

**Authors:** M. M. Kamruzzaman, Ibrahim Alrashdi, Ali Alqazzaz

**Affiliations:** ^1^Department of Computer Science, College of Computer and Information Sciences, Jouf University, Sakakah, Saudi Arabia; ^2^Faculty of Computing and Information Technology, University of Bisha, Bisha, Saudi Arabia

## Abstract

Revolution in healthcare can be experienced with the advancement of smart sensorial things, Artificial Intelligence (AI), Machine Learning (ML), Deep Learning (DL), Internet of Medical Things (IoMT), and edge analytics with the integration of cloud computing. Connected healthcare is receiving extraordinary contemplation from the industry, government, and the healthcare communities. In this study, several studies published in the last 6 years, from 2016 to 2021, have been selected. The selection process is represented through the Prisma flow chart. It has been identified that these increasing challenges of healthcare can be overcome by the implication of AI, ML, DL, Edge AI, IoMT, 6G, and cloud computing. Still, limited areas have implemented these latest advancements and also experienced improvements in the outcomes. These implications have shown successful results not only in resolving the issues from the perspective of the patient but also from the perspective of healthcare professionals. It has been recommended that the different models that have been proposed in several studies must be validated further and implemented in different domains, to validate the effectiveness of these models and to ensure that these models can be implemented in several regions effectively.

## 1. Introduction

The smart city is an emerging concept that is based on the integration of various electronic devices and citizens that enhance the flow of information [1]. Ahvenniemi et al. [2] define smart cities as the ones that have an intelligent, integrated, and cost-effective technology that connects different aspects of the cities like transportation, resource usage, waste management, and human health. These systems are critical in handling the challenges caused by the massive urbanisation of cities that have led to population increase along with issues like traffic congestion, poor health management, crimes, and environmental unsustainability [3]. Thus, smart cities can play a massive role in the improvement of the lives and health of the citizens through advanced management. It is important to note that due to the growth of the cities, it has become very challenging for the city management authorities to cater to the needs of all the citizens, especially their health. The health of the people becomes a serious concern during the pandemic, as it places an increased burden on the conventionally managed healthcare systems. The conventionally used systems in most of the cities all over the world do not have efficient knowledge and information management that makes handling the pandemic hard. Nonetheless, smart cities can enhance these aspects to make pandemic management more convenient. Moreover, smart cities are also defined as Internet of things (IoT)-based information systems that connect different areas of a city like offices, hospitals, transport, homes, and electronic devices.  Figure 1 shows the most important parts of smart cities where smart technologies have been used for agriculture, vehicles, home, education, industries, transport, healthcare, and so on. IoT is an integrated network that helps connect various devices, people, and places. Unlike the conventional Internet that only has a cyber interface, the IoT has a physical interface as well, which comprises devices like sensors. Sensors are one of the most important parts of smart cities and IoT networks as they help gather, process, and transfer information. Thus, these systems are very effective in managing healthcare systems that require efficient coordination between authorities and citizens. The integration of the citizens, hospitals, authorities, and other healthcare elements help the smart cities provide adequate and quick response to the people in need of the desired healthcare services [4]. Also, surveillance is an important part of IoT-based smart cities that make them highly effective in data collection and application of smart strategies. Thus, through the use of different features of smart cities like communication, information management, and surveillance, health risks can be mitigated.

The Internet of Medical Things (IoMT) is a collection of devices that are used in healthcare services and applications that can communicate with the latest communication technologies. By connecting patients to their healthcare professionals and enabling the transmission of health information over a secure communication network, it could help decrease hospital visits as well as the huge burden on medical systems. In 2016, the international IoMT industry was valued at $22.5 billion and it hopes to achieve $72.02 billion by the year 2021, growing at a compound annual rate of 26.2% as per the Frost and Sullivan report. The IoMT industries are equipped with smart electronics devices which are designed solely for health care industries that can be used on the body, or in society, or at home, or at hospital. These devices can provide real-time information such as health conditions, location, and other important information and services [5].

On the other hand, according to the study conducted by the UN, it has been identified that 68% of the overall global population is living in urban regions. Due to the increasing number of patients and limited hospitals, the healthcare industry is facing numerous challenges. Revolution in healthcare can be experienced with the advancement of smart sensorial things, Artificial Intelligence (AI), Machine Learning (ML), Deep Learning (DL), and edge analytics with the integration of cloud computing; and connected healthcare is receiving extraordinary contemplation from the industry, government, and the healthcare communities [6, 7]. Connected Health care combines concepts like mobile communication, digital instruments, 6G, AI-based smart devices, and health management software in which everything is intended to serve the patient needs and also share whatever medical-related information can be shared, thereby helping patients to get medical treatment in the most effective and appropriate manner possible. All parties in this connected healthcare system are “connected” by timely sharing accurate patient information. It is an essential component of the future of healthcare because it aims to ensure that doctors, patients, and family members have access to important information any time. It can be depicted that in this new era, IoMT has provided a broad vision by using smart objects with the processing of massive amounts of complex data to provide the best and multiple services. On the other hand, due to the extensive connectivity of IoT devices to provide frequent connected health services, it can also be considered as a storage burden and computation-intensive at every edge device [8, 9]. This challenge can be addressed by considering that the incorporation of AI and strong edge computation can deliver acquisition of vast complex data and computation services intelligently at edge network for intelligent decision-making that is critical for analysis by professionals [8]. It has been identified that the edges in IoMT can deliver advanced services to the clinicians, caregivers, and physicians from anywhere and at any time without interruption. It has also been identified that the solution provided by the Edge AI is better than the cloud AI [10, 11]. As it does not require connection, cost related to data communication, privacy risk, and power consumption is also reduced as compared to cloud AI. Hence, it can help to develop wearable multifaceted devices that are better at reducing the complexity in healthcare. In addition, responding strategically to complex system data updates can allow healthcare to work smartly [12].

The aim of this study was to conduct a systematic review based on identifying new challenges, opportunities, evaluation of case studies, and applications of Edge-AI for connected healthcare in smart cities. With this, the chances of the implementation of Edge AI in smart cities and for the modernising of the urban regions as smart cities will be increased. The main aim was to find suitable technologies for handling new strains of different diseases, to find new ways of diagnosis and treatment, and to enable the healthcare system to integrate new technology, upgrade the quality of clinical outcomes, and help achieve high patient and physician satisfaction rates. Furthermore, this systematic review discusses some of the past milestones related to these technologies in healthcare systems and discusses promising research directions and their limitations. The selection of the papers for the systematic review is supported by the application of the AMSTAR and PRISMA tools. The review paper is systematically structured. The brief introduction and the background of the study are followed by a comprehensive discussion of the selected methodologies for data collection. After that, the proceeding sections present results of the systematic review, specific findings of the study, and a conclusion that demonstrates the overall outcome of the study.

## 2. Methodology

### 2.1. Data Collection

The present study is based on the qualitative research approach that will allow the researcher to periodically synthesize the relevant literature pertaining to the subject focus of this study. The selection of this research approach is supported by the research philosophy of interpretivism. Thus, this research paradigm emphasises the qualitative study of the research phenomenon rather than quantitative. Moreover, bearing in mind the descriptive character of the present study, the qualitative approach will enable the researcher to review and synthesize a comprehensive amount of the relevant literature. In this regard, the researcher has incorporated a systematic review strategy in pursuit of this objective. Before conducting the evaluation, the review procedure was created. The relevant good quality literature including articles and journals were selected while their findings are reviewed, analysed, and evaluated. Since it has been established that the present study is based on the systematic review of the relevant literature, high-quality journal articles will be identified. It is intended to select the most relevant research articles that will be critically analysed and reviewed. In order to eliminate any kind of bias in the findings, it is imperative to exhaust multiple sources for the acquisition of papers. As per the standards of the AMSTAR, a minimum of two data sources should be used for the extraction of the studies. Secondary data are collected from already published research articles through different search engines including Web of Science, Scopus, PubMed, Google Scholar, and Science Direct.

### 2.2. Inclusion and Exclusion Criteria

It is critical to bear in mind that studies that research studies can be prone to several biases including nonrandomised intervention studies. There are a number of techniques for evaluating the quality of the studies in order to ensure that they are free from biases. In this regard, the two systematic tools stood out among the rest. One of them is the A Measurement Tool to Assess Systematic Reviews (AMSTAR) tool. AMSTAR has been classified as a trustworthy and valid instrument for assessing the methodological quality of a study. The survey comprises eleven questions against which the quality of the papers is assessed in terms of the appropriateness of the techniques used in the papers. For the present study, the AMSTAR tool is incorporated for assessing the quality of the research. The tool assesses the study quality by assessing them against a set of questions. The researcher completed a survey supplied by the tool which then offered to rate the quality. The appendix of the study contains a quality evaluation that was evaluated as “moderate” by the online assessment instrument. AMSTAR assisted in analysing the methodological and the analytical consistency of the findings of the identified articles. The studies published in the last 6 years from 2016 to 2021 are included, whereas the studies published before this period are excluded. Moreover, the studies with ethical issues or those that are not peer-reviewed or have some conflicts are excluded. The selection process is represented through the Prisma flow chart represented in Figure 2.

### 2.3. Review of Relevant Articles

Only peer-reviewed studies and those that included relevant keywords, namely, AI, edge AI, IoT, deep learning, machine learning, smart cities connected healthcare, big data, machine learning, and deep learning, were selected.

### 2.4. Study Selection and Data Abstraction

Due to limited pages, a total of 22 articles are selected which are divided into 2 sections, namely, inclusion of Edge AI and connected healthcare in smart cities. Each section includes 11 studies.

### 2.5. Quality Assessment

In this study, secondary data are collected through relevant studies, after quantitative analysis has been done. The selected studies are systematically reviewed and relevant results are represented in Tables 1 and 2.

## 3. Results

### 3.1. Opportunities, Challenges, and Applications of Edge-AI

According to Pazienza et al. (2019), there are numerous applications of Edge-AI for connected healthcare in smart cities. The edge computing architecture should be addressed so that processing can take place at the gateways (edge nodes) or the devices (end-nodes). It will help in lessening unnecessary processing latency and data traffic, and is significant for applications like critical analysis and monitoring of the patient [13]. For different applications relevant to patient monitoring, the emphasis is placed on developing and designing edge nodes. However, the end-nodes can be differentiated further in a healthcare situation. For example, interactive devices can refer to any stationary hardware or a mobile component that facilitates the interaction between the environment of the user and the human user like wearable devices, speech recognition devices, and smartphones [14]. The ambient devices can refer to any kind of consumer electronics that is categorised by their capability of perceiving at a glance like smart applications, smoke sensors, and motion sensors. Lastly, medical devices can refer to devices to be used for medical purposes, like compensation, alleviation, treatment, monitoring, prevention, and diagnosis of an injury or a disease [13]. Syed et al. (2021) concluded that numerous opportunities can be gained through Edge-AI in smart cities [15]. These opportunities can also be availed by the healthcare sector. A universal synopsis of the state permitting for the usage of big data algorithms of the city can be gained through the data collected by the sensors in IoT systems (Edge-AI) for developing new healthcare services and applications. For the growth of new data science algorithms for service delivery, a great opportunity can be also gained through this heterogeneous data. To make deployment of IoT (Edge-AI) cheaper and easier, there is a huge monetary value toward the usage and development of networking technologies, effective data storage methods, and cheap encryption techniques. For IoT (Edge-AI) in smart cities, another opportunity can also be availed by the development of new sensor technologies. Wider usage and development of IoT (Edge-AI) services may also be contributed by the development of low-cost, effective, and newer sensors [15].

The study by Umair et al. (2021) pointed out that numerous challenges can be faced in the case of Edge-AI for connected healthcare in smart cities [16]. Umair et al. (2021) highlighted more accessible healthcare, AI algorithms on healthcare devices (edge AI), research-grade wearables, energy harvesting wearables, or low-energy as some of the major challenges faced in the healthcare sector [16].

Amin and Hossain (2021) conducted a survey to evaluate the recent and revolutionising frameworks of edge computing, effective technologies for smart healthcare services, challenges and opportunities of different scenarios related to applications [18]. S. U. Amin and Hossain (2021) evaluated edge intelligence which is dedicated to targeting the classifications of health data with the identification and tracking of vital signs by utilising the deep learning technology where billions of edge devices are connected (see Figure 3) [18]. Another purpose of this study was to comprehensively analyse the usage of classification based on cutting edge AI and techniques that can be implemented for edge intelligence. However, it cannot be neglected that challenges related to security and complex computation are associated with Edge AI [18]. The contribution of this study is that it has provided potential recommendations based on research for enhancing the services related to Edge AI computation for healthcare services in smart cities. Along with it, IoT solutions are also highlighted focusing on the edge platform for the growth of the healthcare industry [19].

With the increasing population, several new diseases have emerged like Covid-19 [20]. It has been evaluated that with the implication of a 5g wireless connection based on tactile edge technology, these kinds of pandemic diseases can be controlled [19]. It has been identified that the implication of a hierarchical-edge-based computing system delivers numerous advantages which may include scalability, low latency, and the fortification of model data related to training and allow the researchers to enable the evaluation of COVID-19 with the reliable local edge server [18]. Moreover, the numerous algorithms based on deep learning (DL) face two main challenges which comprise the fact of training a huge dataset and to acknowledge the results with the ethical implications and certification by the healthcare authorities and others [17].

Hossain et al. (2020) conducted a study to propose a B5G model that is based on utilising the 5G network's functionality related to high-bandwidth, low-latency, for detecting the cases of COVID-19 [21]. The results of this framework are based on utilising the images obtained through CT-scan and X-ray; hence, a massive competitive surveillance system is built utilising the thermal cameras and IP surveillance to efficiently monitor the activities related to mask-wearing, body temperature, and social distancing [21]. In the study conducted by Shamim Hossain et al. (2020), 3 different DL models are investigated in the proposed B5G framework including Deep tree, ResNet50, and Inception v3 [21].

For processing and storage of data, it has been analysed that the fog and edge computing models promote smarter and reliable systems without the need of depending on cloud services. A. Nawaz et al. (2019) proposed an Ethereum Blockchain-based framework with Edge AI for analysing the data at the network edge and for keeping track of the parties who are dedicated to access the analytical outcomes, stored in disseminated databases [22]. This framework helped to overcome the challenge of increased security issues due to the addition of new coatings in the network design [22].

S. Tuli et al. (2020) conducted a study to present a vision of implementing a holistic framework that can meet the increasing needs of healthcare and patients [23]. The vision is also based on explaining the conceptual framework which can deliver a profound response to the elevating demands. The presented model is presented with the complete detail of interaction at numerous levels, namely, blockchain, AI, for computing, and machine learning [23]. F. Alshehri and G. Muhammad (2020) conducted a comprehensive survey by including researches conducted from 2014 to 2020 related to IoMT and IoT based on Edge AI to provide smart healthcare services [24, 50]. Results of the study showed that the major challenges of smart health care include device communication, the barrier to information management, security issues, sensors' interoperability, device management, and the use of AI efficiency. It has also been identified that IoMT devices can help to diagnose disease and to reduce illness [25].

According to the qualitative secondary study conducted by H. A. Imran et al. (2020), it has been identified that the main issues related to IT applications may include lack of security, latency, bandwidth, and privacy [26]. From the evaluation of the studies conducted in the last 6 years, it has been identified that approximately 20 million IoT devices will elevate the issues related to sending data to the cloud and processing. Results of the study showed that the increasing challenges can be minimised by the implementation of systems based on data processing on the network nodes and layers which is known as edge computing and fog computing respectively [26].

L. Greco et al. (2020) conducted a review-based study to evaluate the use of IoT for predicting the solutions for connected health care in smart cities. In this paper, solutions are presented from the initial stage of health monitoring feasibility through from wearable sensors to the detailed discussion related to the modern trends in edge and for computing for connected healthcare [27].

Dianlei Xu et al. (2020) pointed out that Edge intelligence aims to improve data processing while protecting the privacy and security of the user's data [28]. Edge caching, edge inference, edge training, and edge offloading are identified as four key components. Researchers also discussed edge intelligence from various perspectives, such as applicable scenarios, performance, methodology, and so on, and summarised their benefits and drawbacks. Five important future research directions and development trends are also discussed in their paper: data scarcity, adaptability of model/algorithms, data consistency, incentive mechanisms, and privacy and security [28].

### 3.2. Opportunities and Challenges for Connected Healthcare in Smart Cities

Connected Healthcare can be defined as a dynamic area of digital health incorporating socio-technical frameworks for efficient delivery and management of healthcare to encourage efficient and significant interventions, services, and designs for the construction of smart cities [29]. Hossain [38] has conducted a study to present a cloud-based smart healthcare monitoring model. This model can effectively interact with the environment, different nearby smart devices, and stakeholders of smart cities for accessible and affordable healthcare [30]. In the case study of healthcare monitoring system, the voice pathology detection is implemented for smart city with two different types of signals. As a result, devices are connected with the Internet, and signals can be transmitted to the cloud using the three-tier architecture for Edge-AI-based connected healthcare systems, as shown in Figure 4. After processing, the signals are classified into pathologic and normal along with a confidence score. The outcomes are sent to healthcare professionals to help them in taking the right decision. After evaluating the results, it has been identified that the presented method is found to be successful in achieving VPD, with an accuracy of 93% [30].

It has been identified that using social media for communication related to healthcare is affected by the issues related to confidentiality, data deluge, limited reliability, privacy, and quality. The filtering mechanism is found to fail due to duplicate or similar questions [31]. A. Kumar (2020) proposed a hybrid deep learning model to overcome the issue of semantic question matching for identical question couple recognition. After evaluating the results, it has been identified that the proposed model has shown an accuracy of 86.375% [32].

It has been identified that the latest IoT systems are dependent on semantic web technology for the integration of the data and for ensuring the interoperability of the web services. It has been identified that there is a huge literature gap present related to ensuring semantic interoperability in IoT-based systems [32]. Gyrard, Amelie et al. (2016) conducted a study to analyse the most acceptable semantic-based IoT approaches for recognising the main necessities deterring IoT-semantic interoperability [33]. Gyrard, Amelie et al. (2016) proposed an SEG 3.0 methodology to amalgamate, associate, and offer semantic interoperability [33]. The proposed methodology is applied to the Internet of Things (IoT) including different case studies based on smart cities including “the M3 model for assisting designers in scheming the semantic-based IoT applications,” the “FIESTA-IoT-EU project especially for IoT-semantic interoperability,” and the “VITAL EU project,” especially for smart cities. It has been identified that this methodology can be used anywhere in different domains present in smart cities with the main advantage of incorporating the heterogeneous data by supplementing the value in it [34].

Studies have highlighted that in smart cities, it is mandatory now to have an effective, secure, and accessible healthcare system for the citizens [35]. G. Tripathi et al. (2020) conducted a study where they have discussed numerous elements of technology that can be incorporated in healthcare and can present a secure and effective “Smart Medical System” model for the ecosystem of smart cities [36]. This study encourages real-time analysis and presents the concept of “mobile edge computing” that is found to be secured for critical edge computations. This framework is based on using the concept of blockchain to protect the data of medical patients. Through this, it became possible to demonstrate the ways through which the big and complex medical data can be stored by using IoT sensors and devices [36].

M. I. Pramanik (2017) conducted a study to evaluate numerous complex data in different domains in healthcare by utilising smart system technology and for critical analysis of the state-of-art progressive healthcare industry [37]. In this study conducted by M. I. Pramanik (2017), the evaluation of several big and complex data in the context of healthcare is processed by proposing a conceptual framework known as “Big data-enabled Smart Healthcare System Framework” [37]. The results of the study can be used by healthcare systems to reinforce the strategic organisation of smart systems and complex data in the healthcare context [37].

A. Alghamdi et al. (2021) conducted a study to present a computer-aided diagnosis system for detecting motor imagery signals by utilising the convolution neural network in smart cities, especially for urban healthcare [53]. In this study, 2 different transfer learning methods are used for retraining the VGG-Net and gained 2 different networks which include VGG-MI-1 and VGG-MI-2 [53]. In the 1st proposed model, the final layer of the model is substituted with a particular layer as per the optimisation of numerous functions to condense overfitting. In the 2nd proposed model, the 1st layer of the model is designated as the prompt feature of the images obtained through ECG for defining it with revealing topographies [53]. Results of the study showed that the VGG-MI-1 showed sensitivity, specificity, and accuracy of 98.76%, 99.17%, and 99.02%, respectively, and the VGG-MI2 model showed sensitivity, specificity, and accuracy of 99.15%, 99.49%, and 99.22%, respectively [53]. A. N. Navaz (2021) conducted a study to evaluate the challenges in connected healthcare in smart cities. For this, they have focused on the latest challenges in Covid-19 which is a global issue in recent years [39]. In this study, the related cases are reflected to evaluate how many states have tackled this pandemic situation successfully by incorporating the latest advanced technology including the processing of big data, mobile applications, artificial intelligence, Internet of Things, cloud computing, blockchain, and robotics. It has been identified that Smart and Connected Health (SCH) is an effective solution for overcoming the increasing challenges faced by the healthcare industry [40].

M. Poongodi et al. (2021) conducted a study to explore the implication of the latest trends in connected healthcare including IoT and 5g wireless connection [41]. In this study, M. Poongodi et al. (2021) highlighted the issues faced by patients related to the service of an ambulance in emergency cases [41]. After evaluating the literature review, it has been identified that the ambulance tracking system and patient monitor can be used effectively for quick diagnosis by using the data of breath rate, temperature, and heartbeat [40]. These details can be sent directly to the hospital or doctor from an ambulance to save time in diagnosis through a wireless 5G connection [41]. Moreover, an instant touch button can be provided to the patient which he or she will press in case of emergency to call or send a short quick message instantly to the hospital or any relative; hence, the life of the patient can be saved from several risks. With the android application and IoT sensors, ambulances can also be tracked so that the hospital staff can become ready to deal with patients [41].

Diagnosis of COVID-19 using Chest X-ray Images using synergic deep learning (SDL) is proposed for smart healthcare system [42]. Authors have shown that classification of COVID-19 can be effectively performed by the integration of FBL and SDL. Simulation with different datasets is conducted for ensuring the effectiveness of the FBF-SDL model over the existing models and to examine the classifier outcome of the SDL model [42]. In this paper, authors created a new synergic DL-based COVID-19 classification model with Chest X-ray images. To improve the quality of the chest X-ray images, the SDL model undergoes initial processing using the FBF technique [42].

After evaluating the previous literature, it has been identified that urban health is limitedly explored; hence, IoT devices can be used to measure the data for smart homes with fog and cloud computing [51]. S. Nosratabadi et al. (2019) conducted a study to explore various aspects of smart cities [25]. They have presented deep learning and machine learning methods. The reason behind using these methods is to help advance the models concerning uncertainty analysis, and planning and prediction of urban development and smart cities. Results of the study showed that a total of 5 machine learning and deep learning methods are found to address various aspects of smart cities. These methods include deep learning; artificial neural networks; ensembles, hybrids, neuro-fuzzy, and Bayesians; support vector machines; and decision trees. Through novel taxonomy, in this study, the advancement related to the development of the model and related application domains are presented specifically for smart cities and urban sustainability [25, 43].

## 4. Discussion

### 4.1. Recent Development

In this era of modern technology, the installation of smart healthcare systems is required to satisfy the needs of individual patients and to assist healthcare professionals to provide better diagnosis and treatment opportunities [44]. With the integration of IoT sensors, 5G, and AI-edge computing, it has become easy to provide better healthcare real-time solutions along with encouraging privacy, satisfying latency criteria, reducing cost, and energy consumption [45]. Several countries have used Smart and Connected Healthcare for diagnosis, detection, tracking, monitoring, resources allocation, and controlling. It has also been used for monitoring, tracking, controlling, and resource allocation. After evaluating several search studies, it has been evaluated that for the economic growth of the country, Smart Cities play a significant role. Not only this, but they also play a significant role to enhance the welfare of the citizens. They also help to enhance the capability of the citizens to use technology for building sustainable services. It has been identified that for building smart cities, computational methods play a major role. The reason behind this is that these methods are the building blocks of decision-making. They assist in making policies and provide the best services for the people. J. T. de Souza et al. (2019) conducted a study to represent a systematic review related to approaches of machine learning and data mining that can be adopted for the development of smart cities [35]. A total of 39 articles were evaluated for analysing the data mining and machine learning techniques. After evaluation, it has been found that predictive analysis is the most used technique, focusing mainly on the areas of smart environment and smart mobility. Hence, through this study, it can be suggested that the government authorities can use such approaches for the development of smart cities that are also necessary to help in the achievement of Sustainable Development Goals [25, 35]. Furthermore, still, there are several challenges present related to its validation and detailed research to be used all over the world [39].

### 4.2. Opportunities

From the literature review, it has been evaluated that the Edge-AI and related technology and domains including IoT, Big Data processing, Internet of Medical Things (IoMT), Edge learning, 5g, 6g, etc., [32]. have provided impressive advancement in several domains, especially in healthcare, and saved the lives of thousands of people. With the increasing population, several new diseases have emerged like Covid-19. It has been evaluated that with the implementation of advanced technology, this kind of pandemic disease can be controlled. With edge AI, diagnosis has become easy [13]. To illustrate, at the hospital edge nodes, a CT scan can perform the diagnosis effectively and provide accurate results. From the results of the study, it has been identified that AI has shown a massive contribution for resolving the healthcare issues including dealing with emerging diseases, diagnosis, and treatment of new variants, processing of complex data, better accuracy in outcomes, high sensitivity and advanced control, and tracking and monitoring [40].

### 4.3. Challenges

It can be depicted that, in this new era, the IoT has the ability of processing of massive amounts of complex data to provide the best services. On the other hand, due to the extensive connectivity of IoT devices to provide frequent connected health services, it is also considered as a storage burden and computation-intensive at every edge device [8]. This challenge can be addressed by considering that the incorporation of AI and strong edge computation can deliver acquisition of huge complex data and computation services intelligently at edge network for intelligent decision-making that is critical for analysis by professionals [9]. It has been identified that the edge-IoT services can deliver an advanced experience to the clinicians, caregivers, and physicians from anywhere and at any time without interruption. It has also been identified that the solution provided by Edge AI is better than the cloud [9]. It has been identified that the previous studies did not primarily focus on fog and cloud computing architecture, authentication, security, sensor type, and devices that can be used effectively in the frameworks of edge computing [33]. Hence, it has been required to focus on the applications of IoT and Edge AI in healthcare. One of the major challenges is to implement such systems by converting urban areas into smart cities which require detained research and funding. Through literature, it has been identified that several factors are involved that can negatively impact the adoption of Edge AI. Hence, it is required to conduct further research to overcome the negative impacts of such factors [46].

### 4.4. Future Work

It has been recommended that different models have been proposed in several studies as discussed in this study; hence, these models must be validated further and implemented in different domains to validate the effectiveness of these models and to ensure that these models can be implemented in several regions effectively [47]. The main issues identified in the healthcare systems is the late diagnosis, wrong treatment, and misinterpretation due to which it is required that the proper systems must be installed with the incorporation of advanced software, tools, and technologies [25]. For the utilisation of artificial intelligence effectively for the construction of Smart Cities, it is required that the available data be evaluated and stored so that it can be used for making effective algorithms of AI and deep learning for the betterment of healthcare systems and patients' health [48]. For the better future of the healthcare system, 6 key areas are required to give proper attention and detailed research including interoperability, data sharing, behavior change, scientific breakthrough, and empowered consumers [41]. By focusing on these areas, the chances of successfully transforming the present healthcare system from treatment centres to well-being and diseases prevention centres are high. In addition, the urban population requires more attention. They have limited access to healthcare; hence, limited data are available. Therefore, it is essential to facilitate and educate such populations so that their basic healthcare needs can be fulfilled and the mortality rate can be reduced in such areas due to the pandemic situation, resource scarcity, and inefficient treatment plans [49]. Advanced networking solutions are required to be implemented so that effective communication can be made at distant locations to resolve issues and guide the patients with their issues. It is required to implement advanced communication technologies with fast networking devices so that the issues related to healthcare concerns can be avoided. There is limited research available related to the implementation and effectiveness of connected healthcare in smart cities; therefore, further research must be conducted so that the related concerns can be clarified and effectiveness can be validated by minimising the related challenges identified in this study.

## 5. Conclusion

Edge-AI and IoMT are the advanced technologies that are being currently used in various parts of connected healthcare in Smart Cities. The use of these technologies in the monitoring and management of connected healthcare can also prove to be very beneficial as they can reduce the required human efforts and improve the efficiency of management. In this study, a systematic review has been performed to identify the challenges, opportunities, and applications in Edge AI for connected healthcare in Smart Cities. Several studies are reviewed systematically divided into 2 sections. After evaluating the selected studies, it has been identified that with increasing population and disease spread, it has become increasingly difficult for the healthcare professionals to manage the patient data; to respond to the queries of patients; to handle the emergency cases; to track patient history; to monitor, track, and evaluate patients; and to diagnose and treat different diseases which are reacting differently in patients. However, it has been identified that these increasing challenges can be overcome by the implementation of Edge AI, IoMT, 5G, fog, and cloud computing. Still, limited areas have implemented these latest advancements and also experienced improvements in the outcomes. These implementations have shown successful results not only in resolving the issues from the perspective of the patient but also from the perspective of healthcare professionals. It has been recommended that the different models have been proposed in several studies; hence, these models must be validated further and implemented in different domains to validate the effectiveness of these models and to ensure that these models can be implemented in several regions effectively [52].

## Figures and Tables

**Figure 1:** Smart city concept [25].

**Figure 2:** PRISMA process.

**Figure 3:** Design of IoI-based healthcare system [18].

**Figure 4:** Three-tier architecture for Edge-AI-based connected healthcare systems.

**Table 1:** Summary of Findings of the Selected Studies based on Edge-AI.

No	References	Study design	Objectives	Findings	Limitations
1	Amin and Hossain (2021) [18]	Qualitative analysis	To evaluate the recent and revolutionising frameworks of edge computing, effective technologies for smart healthcare services, the challenges and opportunities of different scenarios related to applications. To comprehensively analyse the usage of classification based on cutting edge AI and techniques that can be implemented for edge intelligence	The contribution of this study is that it has provided potential recommendations based on research for enhancing the services related to Edge AI computation for healthcare services in smart cities. Along with it, IoT solutions are also highlighted focusing on the edge platform for the growth of the healthcare industry	A limited number of researchers are available

2	Syed et al. (2021) [15]	Qualitative analysis	To provide holistic coverage of the Internet of Things in Smart Cities. To review the most prevalent applications and practices in different domains of Smart City. To examine the challenges of adopting IoT systems for smart cities along with mitigation measures	Broad coverage of IoT in Smart Cities is presented as an important enabling of smart city services. The privacy and security issues faced by IoT also have been discussed in detail	Different research methods could have been used for making DL (deep learning) and ML (machine learning) more explainable further

3	Umair et al. (2021) [16]	Qualitative analysis	Impact of covid-19 on the adoption of IoT	Identified the challenges that are needed to be addressed	Further research is required

4	Amin and Hossain (2021) [18]	Qualitative analysis— survey	To evaluate the recent and revolutionising frameworks of edge computing, effective technologies for smart healthcare services, the challenges and opportunities of different scenarios related to applications. To comprehensively analyse the usage of classification based on cutting edge AI and techniques that can be implemented for edge intelligence	The contribution of this study is that it has provided potential recommendations based on research for enhancing the services related to Edge AI computation for healthcare services in smart cities. Along with it, IoT solutions are also highlighted focusing on the edge platform for the growth of the healthcare industry	A limited number of researchers are available

5	Hossain et al. (2020) [21]	Quantitative study—experiment design	To propose a B5G model that is based on utilising the 5G network's functionality related to high bandwidth, low latency, for detecting the cases of COVID-19	The framework was found to efficiently monitor the activities related to mask-wearing, body temperature, and social distancing	Only 3 DL models are used and the framework is required to be tested in future with the protease sequence analysis

6	Nawaz et al. (2019) [22]	Quantitative study—cross-sectional study design	To propose an Ethereum Blockchain-based framework with edge AI	It helped to overcome the challenge of increased security issues due to the addition of new coatings in the network design	Cause-and-effect relationship is not presented due to the nature of the study design

7	S. Tuli et al. (2020) [23]	Qualitative study design	To present a vision of implementing a holistic framework that can meet the increasing needs of healthcare and patients	The model helped to identify challenges, opportunities, and current trends in the healthcare industry,.	Used limited deep learning techniques to predict failures

8	F. Alshehri and G. Muhammad (2020) [24]	Qualitative study design— a comprehensive survey	To evaluate the studies based on IoT, medical signals, IoMT, AI-edge, and cloud services	The major challenges of smart health care are identified, which includes device communication, the barrier to information management, security issues, sensors' interoperability, device management, and use of AI efficiency. It has also been identified that IoMT devices can help to diagnose disease and to reduce illness	Researches conducted after 2020 are not included

9	A. Imran et al. (2020) [26]	Qualitative study design— secondary literature review	To evaluate the studies based on edge computing and fog computing	Increasing challenges can be minimised by the implication systems based on data processing on the network nodes and layers which is known as edge computing and fog computing, respectively	Researches conducted after 2020 are not included

10	L. Greco et al. (2020) [27]	Qualitative study design— secondary literature review	To evaluate the studies based on providing solutions to the smart healthcare services through edge computing and fog computing	Presented solutions from the initial stage of health monitoring feasibility through from wearable sensors till the detailed discussion related to the modern trends in edge and for computing for connected healthcare	Researches conducted after 2020 are not included

11	Dianlei Xu, Tong Li, Yong Li, Xiang Su, Sasu Tarkoma, Tao Jiang, Jon Crowcroft, Pan Hui (2020) [28]	Review-based qualitative study	To conduct a review on Edge intelligence	Edge caching, edge inference, edge training, and edge offloading are identified as four key components	Researchers also discussed edge intelligence from various perspectives, such as applicable scenarios, performance, methodology, and so on, and summarised their benefits and drawbacks.

**Table 2:** Summary of Findings of the Selected Studies based on connected healthcare in Smart Cities.

No	References	Study design	Objectives	Findings	Limitations
1	Hossain (2017) [18]	Quantitative study	To present a cloud-based smart healthcare monitoring model to effectively interact with the environment, different nearby smart devices, and stakeholders of smart cities for accessible and affordable healthcare	The presented method is found to be successful in achieving VPD, with an accuracy of 93%	Further research is required to validate the results and to increase the model accuracy

2	A. Kumar (2020) [32]	Quantitative study	To propose a hybrid deep learning model to overcome the issue related to the filtration of duplicated questions in healthcare	The proposed model has shown an accuracy of 86.375%	Further research is required to validate the results and to increase the model accuracy

3	Gyrard, Amelie et al. (2016) [33]	Qualitative study	Proposed an SEG 3.0 as a methodology	Proposed an SEG 3.0 methodology to amalgamate, associate, and offer semantic interoperability	The proposed methodology was not implemented in other domains

4	G. Tripathi et al. (2020) [36]	Qualitative study	To encourage real-time analysis and to present the concept of “mobile edge computing”	The proposed model is found to be secure for executing time-bound and critical edge computations	Further research is required to use this model in healthcare systems

5	M. I. Pramanik (2017) [37]	Qualitative study	To propose a conceptual framework known as “big data–enabled smart healthcare system framework”	The results of the study can be used by healthcare systems to reinforce the strategic organisation of smart systems and complex data in the healthcare context	The framework is not practically implemented in the healthcare industry; hence, research is required to validate the results first for actual implementation

6	A. Alghamdi et al. (2021) [53]	Quantitative study	To use 2 different transfer learning methods for retraining the VGG-Net and gained 2 different networks which include VGG-mi-1 and VGG-mi-2	Results of the study showed that the VGG-MI-1 showed sensitivity, specificity, and accuracy of 98.76%, 99.17%, and 99.02%, respectively, and the VGG-MI2 model showed sensitivity, specificity, and accuracy of 99.15%, 99.49%, and 99.22%, respectively	The effectiveness of the model is validated only for ECG data

7	A. N. Navaz (2021) [39]	Review-based qualitative study	To conduct a review on smart and connected health (SCH)	Several countries have used SCH successfully for diagnosis, detection, tracking, monitoring, resources allocation, and controlling of the Covid-19 cases	There are several challenges present related to its validation and detailed research to be used all over the world

8	M. Poongodi et al. (2021) [41]	Review-based qualitative study	To explore the implication of the latest trends in connected healthcare including IoT and 5g wireless connection	IoT and 5g wireless connection can be used effectively to reduce the challenges faced by patients and the healthcare profession also in an emergency	These systems are required to validate further in real-time applications

9	Nosratabadi et al. (2019) [25]	Review-based qualitative study	To explore the needs of the extraction of big data urban population	The exploration of urban data found to be helpful to provide a key to supplement a contemporary notion of Big Data for reaching the aim of sustainable and resilient smart cities as figured out in the 11th Sustainable Development Goal	Different datasets are not compared; hence, further research is required

10	Hossain, Muhammad, and Alamri (2017) [30]	Qualitative study	To represent the state-of-the-art of deep learning and machine learning methods that can be used in real time	Results of the study showed that the identified deep learning and machine learning methods mainly addressed the issues in the main domains including urban transport, health, and energy	Deep learning and machine learning methods are found to be effective in specific domains; hence, research is required to explore every domain deeply

11	K. Shankar et al. (2021) [42]	Qualitative study	Diagnosis of COVID-19 using chest X-ray images using synergic deep learning (SDL) is proposed for smart healthcare system	The integration of FBL and SDL resulted in the effective classification of COVID-19. To investigate the classifier outcome of the SDL model, a detailed set of simulations takes place and ensures the effective performance of the FBF-SDL model over the compared methods. Authors have shown that the classification of COVID-19 can be effectively performed by the integration of FBL and SDL. Simulation with different dataset is conducted for ensuring the effectiveness of the FBF-SDL model over the existing models and to examine the classifier outcome of the SDL model	In this paper, authors created a new synergic DL-based COVID-19 classification model with chest X-ray images. To improve the quality of the chest X-ray images, the SDL model undergoes initial processing using the FBF technique. Hence, research is required to explore every domain deeply

**Table 3:** AMSTAR Results,

Blockchain IoT and fog computation for the healthcare services in smart cities' moderate quality review	
1. Did the research questions and inclusion criteria for the review include the components of PICO?	Partially yes
2. Did the report of the review contain an explicit statement that the review methods were established prior to the conduct of review and did the report justify any significant deviation from the protocol?	Yes
3. Did the review authors explain the selection of the study designs for inclusion in the review?	Yes
4. Did the review authors include the comprehensive literature search strategy?	Yes
5. Did the review authors perform the study selection in duplicate?	Yes
6. Did the review authors perform data extraction in duplicate?	Yes
7. Did the review authors justify the exclusion?	Yes
8. Did the review authors describe the included studies in adequate detail?	Yes
9. Did the review authors use a satisfactory technique for assessing the risks of bias in individual studies that were included in the review?	Partially yes
10. Did the review authors report on the source of funding for the studies included in the review?	Yes
11. Did the review authors report any potential sources of conflict of interest including funding they received for conducting the review?	No conflict reported

## Data Availability

The data supporting the findings of this work are available within the article.

## Appendix

AMSTAR Results (Table 3).
